# MicroRNA-138 acts as a tumor suppressor in non small cell lung cancer via targeting YAP1

**DOI:** 10.18632/oncotarget.9480

**Published:** 2016-05-19

**Authors:** Ling Xiao, Hui Zhou, Xiang-Ping Li, Juan Chen, Chao Fang, Chen-Xue Mao, Jia-Jia Cui, Wei Zhang, Hong-Hao Zhou, Ji-Ye Yin, Zhao-Qian Liu

**Affiliations:** ^1^ Department of Clinical Pharmacology, Xiangya Hospital, Central South University, Hunan 410078, P.R. China; ^2^ Institute of Clinical Pharmacology, Central South University, Hunan Key Laboratory of Pharmacogenetics, Changsha, Hunan 410078, P.R. China; ^3^ Department of Histology and Embryology, School of Basic Medical Sciences, Central South University, Changsha, Hunan 410013, P.R. China; ^4^ The Affiliated Cancer Hospital, XiangYa School of Medicine, Central South University, Changsha, Hunan 410014, P.R. China

**Keywords:** non small cell lung cancer, microRNA-138, Yes-associated protein 1, growth, metastasis

## Abstract

MicroRNA (miR)-138 was found to have suppressive effects on the growth and metastasis of different human cancers. In this study, we aimed to investigate the regulatory mechanism of miR-138 in non-small cell lung cancer (NSCLC). We applied the Quantitative real-time PCR (qRT-PCR) to detect the miR-138 levels in NSCLC tissues (n=21) and cell lines, Bioinformatical predication, luciferase reporter assay and western blot to identify the target gene of miR-138. We also applied Cell transfection, MTT, transwell, and wound healing assays to reveal the role of miR-138 in NSCLC cell proliferation and malignant transformation. We observed that miR-138 expression level was significantly decreased in NSCLC tissues compared to their matched adjacent normal tissues. It was also downregulated in tissues with poor differentiation, advanced stage or lymph nodes metastasis, as well as in several NSCLC cell lines compared to normal lung epithelial cell. We further identified YAP1 as a direct target gene of miR-138, and observed that the protein level of YAP1 was negatively mediated by miR-138 in NSCLC A549 cells. Moreover, overexpression of miR-138 significantly inhibited A549 cell growth, invasion and migration, while knockdown of miR-138 enhanced such capacities. Further investigation showed that the cell proliferation capacity was higher in the miR-138+YAP1 group, when compared with that in the miR-138 group, suggesting that overexpression of YAP1 rescued the suppressive effects of miR-138 upregulation on NSCLC cell proliferation. However, we found no difference of cell invasion and migration capacities between miR-138+YAP1 group and miR-138 group. Finally, YAP1 was markedly upregulated in NSCLC tissues compared to their marched adjacent normal tissues. Its mRNA levels were reversely correlated with the miR-138 levels in NSCLC tissues. In summary, our study suggests that miR-138 may play a suppressive role in the growth and metastasis of NSCLC cells partly at least by targeting YAP1.

## INTRODUCTION

Lung cancer is the leading cause of cancer death worldwide, and its incidence has been increasing in recent decades [1]. Therefore, as the most common lung cancer, non-small cell lung cancer (NSCLC) terribly threatens to human health. Despite improvements in diagnosis and combined treatments including surgical resection, radiotherapy and chemotherapy, the overall survival for NSCLC patients still remains poor [2]. Investigations in recent years revealed that deregulation of oncogenes and tumor suppressors played key role in the development and progression of NSCLC [3–5]. Therefore, studies on the regulatory mechanisms of these oncogenes and tumor suppressors should help improve the diagnosis and treatment for NSCLC.

MicroRNAs (miRs), 18-25 nucleotides in length non-coding RNAs, have been demonstrated to act as negative regulators of gene expression through directly binding to the 3′-untranslational region (UTR) of their target mRNAs, leading to either inhibition of their translation or induction of their degradation [6]. Overexpression or downregulation of specific miRs has recently been reported in a variety of human malignancies. Among these miRs, miR-138 generally acts as a tumor suppressor in different cancer types, such as ovarian cancer [7], glioblastoma [8], squamous cell carcinoma [9], head and neck squamous cell carcinoma [10], as well as NSCLC [11]. Overexpression of miR-138 induced radiosensitization in lung cancer cells via targeting SENP1 [11]. Zhang *et al.* demonstrated that miR-138 inhibited the tumor growth of NSCLC via targeting EZH2 [12]. As one miR have many target genes [13], whether other target genes of miR-138 exist in NSCLC still remains to be studied.

Yes-associated protein 1 (YAP1) is a downstream nuclear effector of the Hippo signaling, which is involved in development, growth, repair, and homeostasis. Moreover, as a transcriptional regulator of Hippo signaling, YAP1 was recently found to promote the development and progression of various cancers, and may function as a potential target for the treatment of NSCLC. However, the regulatory mechanism of YAP1 expression in NSCLC remains largely unknown.

In the present study, we aimed to explore the expression levels of miR-138 and its clinical significance in NSCLC. We also studied the molecular mechanism by which miR-138 mediated the growth and metastasis of NSCLC cells involving YAP1.

## RESULTS

### MiR-138 is downregulated in NSCLC tissues and cell lines

To study the role of miR-138 in NSCLC, we examined the miR-138 levels in 21 cases of NSCLC tissues and their matched adjacent non-tumor tissues. As indicated in Figure 1A, most NSCLC showed a decrease in miR-138 expression. Statistical analysis showed that miR-138 expression level was significantly reduced in NSCLC tissues compared to their matched adjacent non-tumor tissues (Figure 1B). Moreover, we found that the expression of miR-138 was significantly lower in poor differentiated NSCLC tissues compared to well/moderate differentiated NSCLC tissues (Supplementary Figure S1A). Besides, NSCLC with higher stage or lymph nodes metastasis also showed significant downregulation of miR-138 expression (Supplementary Figure S1B and S1C). However, its expression seemed not be associated with age, gender or tumor size (Supplementary Figure S1D-S1F). These data suggest that downregulation of miR-138 may contribute to the malignant progression of NSCLC.

**Figure 1:** **A.** and **B.** Real-time RT-PCR was conducted to examine the expression levels of miR-138 in 21 cases of NSCLC and their matched adjacent non-tumor tissues (Adjacent). ** P < 0.01 vs adjacent. **C.** Real-time RT-PCR was conducted to examine the expression levels of miR-138 in four common human NSCLC cell lines, A549, SK-MES-1, H460, and SPC-A1, as well as in a normal human lung epithelial cell line BEAS-2B. ** P < 0.01 vs. BEAS-2B. NSCLC: non-small cell lung cancer.

We further determined the miR-138 levels in four common human NSCLC cell lines, SK-MES-1, A549, H460, and SPC-A1, as well as in a normal human lung epithelial cell line BEAS-2B. As shown in Figure 1C, miR-138 was significantly downregulated in NSCLC cell lines compared to BEAS-2B cells. These data indicated that miR-138 is downregulated in NSCLC.

### MiR-138 shows suppressive effects on NSCLC cell growth and metastasis

Owing to its lowest expression of miR-138 among four NSCLC cell lines (Figure 1C), A549 cell line was selected in later study [14]. To further investigate the role of miR-138 in the regulation of NSCLC cell proliferation, invasion and migration. A549 cells were transfected with miR-138 mimic or inhibitor, then miR-138 level was examined using real-time RT-PCR. As demonstrated in Figure 2A, cells transfected with miR-138 mimic showed a significant increase in miR-138 level, while transfection of miR-138 inhibitor remarkably suppressed the miR-138 level, compared to the control group. MTT assay showed that overexpression of miR-138 significantly inhibited A549 cell proliferation, while knockdown of miR-138 enhanced A549 cell proliferation (Figure 2B), suggesting that miR-138 has a suppressive effect on NSCLC cell growth. Transwell assay and wound healing assay further indicated that overexpression of miR-138 significantly suppressed the invasion and migration of A549 cells, while knockdown of miR-138 enhanced A549 cell invasion and migration (Figure 2C and 2D), suggesting that miR-138 plays an inhibitory role in NSCLC cell metastasis.

**Figure 2:** **A.** Real-time RT-PCR was conducted to examine the expression levels of miR-138 in NSCLC A549 cells transfected with miR-138 mimic or inhibitor, respectively. **B.** MTT assay, **C.** transwell assay and **D.** wound healing assay were further conducted to examine the cell proliferation, invasion and migration, respectively. Non-transfected cells were used as blank control. ** *p* < 0.01 vs. control. NC: negative control.

### YAP1 is a direct target of miR-138 in NSCLC A549 cells

Next, we performed bioinformatic analysis to predicate the putative targets of miR-138, and found that YAP1 might be a target gene of miR-138 and the target site located in the 3′-UTR (Figure 3A). To verify this bioinformatic predication, the wild type or mutant type of YAP1 3′-UTR was constructed and inserted into the psiCHECK-2 vector (Figure 3B). Luciferase reporter assay was then performed in NSCLC A549 cells. As shown in Figure 3C, the luciferase activity was significantly downregulated only in NSCLC A549 cells co-transfected with miR-138 mimic and wild type of YAP1 3′UTR; however, it was unchanged in other groups compared to the control group. These data indicate that YAP1 is a target gene of miR-138 in NSCLC cells. To further confirm this result, we examined the effects of miR-138 on YAP1 expression in NSCLC A549 cells. The protein level of YAP1 was then examined in A549 cells transfected with miR-138 mimic or inhibitor. As shown in Figure 3D, the protein level of YAP1 was significantly reduced in miR-138-overexpressing A549 cells, but markedly increased after knockdown of miR-138, compared to the control group. Based on these data, we demonstrate that miR-138 negatively regulates the protein expression of YAP1 in A549 cells via directly binding to the 3′-UTR of its mRNA.

**Figure 3:** **A.** Bioinformatical predication showed that YAP1 was a putative target gene of miR-138. **B.** The wild type (WT) or mutant (MT) of YAP1 3′-UTR was constructed and inserted into the psiCHECK-2 vector. **C.** A549 cells were co-transfected with wildtype or mutant YAP2 3′-UTR constructs and miR-138 mimic, or scramble miR mimic. Dual-luciferase reporter assay system was used to determine the luciferase activities 48 h after co-transfection. Renilla luciferase activity was normalized to firefly luciferase activity. **D.** Western blot was conducted to examine the protein levels of YAP1 in A549 cell transfected with miR-138 mimic or inhibitor, respectively. Non-transfected cells were used as Control. ** *p* < 0.01 vs. control. WT: wildtype, MT: mutant, NC: negative control.

### YAP1 is involved in miR-138-mediated NSCLC cell growth but not in metastasis

Based on the above data, we speculated that YAP1 might be involved in miR-138-mediated NSCLC cell growth and metastasis. To verify our speculation, miR-138-overexpressing A549 cells were further transfected with YAP1-overexpressing plasmid, in order to rescue the suppressive effect of miR-138 upregulation on YAP1 expression. We found that the protein level of YAP1 was higher in the miR-138+YAP1 group, when compared with that in the miR-138 group (Figure 4A). After that, we determined the cell proliferation, invasion and migration in each group. MTT assay showed that the cell proliferation capacity was higher in the miR-138+YAP1 group, when compared with that in the miR-138 group (Figure 4B), suggesting that overexpression of YAP1 rescued the suppressive effects of miR-138 upregulation on NSCLC cell proliferation. However, as indicated in Figure 4C and 4D, there was no significant difference in cell invasion and migration between the miR-138+YAP1 group and the miR-138 group, suggesting that the suppressive effects of miR-138 on NSCLC cell metastasis was independent with YAP1. In summary, we suggest that YAP1 is involved in miR-138-mediated NSCLC cell growth but not metastasis.

**Figure 4:** **A.** Western blot was conducted to examine the protein levels of YAP1 in A549 cell transfected with miR-138 mimic (miR-138), or co-transfected with miR-138 mimic and YAP1 overexpression plasmid (miR-138+YAP1). **B.** MTT assay, **C.** transwell assay and **D.** wound healing assay were conducted to determine the cell proliferation, invasion and migration, respectively. Non-transfected cells were used as Control. ** *p* < 0.01 vs. miR-138.

### YAP1 is upregulated in NSCLC, reversely correlated with the miR-138 levels

We then examined the mRNA level of YAP1 in NSCLC tissues and their matched adjacent normal tissues. As shown in Figure 5A, 74.1% (20/27) cases of NSCLC showed an increase in YAP1 mRNA expression. Also, its mRNA levels were significantly upregulated in NSCLC tissues compared to their matched adjacent non-tumor tissues (Figure 5B). Moreover, we observed a reverse correlation between the mRNA levels of YAP1 and miR-138 in NSCLC tissues, which further suggests that upregulation of YAP1 may due to the downregulation of miR-138 in NSCLC.

**Figure 5:** **A.** and **B.** Real-time RT-PCR was conducted to examine the mRNA levels of YAP1 in 21 cases of NSCLC and their matched adjacent non-tumor tissues (Adjacent). **C.** The mRNA level of YAP1 was reversely correlated with the miR-138 levels in NSCLC tissues. * P < 0.05 vs. adjacent.

## DISCUSSION

*Zhang et al*. reported that miR-138 was downregulated in NSCLC cell lines and some clinical samples [12]. On account of the small sample size, we detected miR-138 expression in another independent population and several lung cancer cell lines, and investigated the clinical significance of miR-138. In the present study, our data showed that the expression level of miR-138 was frequently and significantly reduced in lung cancer cells and tissues. Moreover, NSCLC tissues with poor differentiation, advanced stage or lymph nodes metastasis showed significant downregulation of miR-138 expression. We observed that miR-138 could inhibit the proliferation, invasion and migration of NSCLC A549 cells. Furthermore, YAP1 was identified as a target gene of miR-138. Moreover, the cell proliferation capacity was higher in the miR-138+YAP1 group, when compared with that in the miR-138 group, suggesting that overexpression of YAP1 rescued the suppressive effects of miR-138 upregulation on NSCLC cell proliferation. However, we found no difference of cell invasion and migration capacities between miR-138+YAP1 group and miR-138 group. Finally, we observed a significant upregulation of YAP1 in NSCLC tissues compared to their matched normal tissues, as well as a reverse correlation between YAP1 and miR-138 levels in NSCLC tissues. Therefore, we suggest that miR-138 inhibits the growth of NSCLC cells partly at least via targeting YAP1.

MiR-138 has been reported to plays a suppressive or promoting role in different human cancers [10, 15, 16]. For example, Yang *et al.* showed that miR-138 could inhibit lung cancer cell proliferation and colony formation, and was associated with radio-sensitization by targeting Sentrin/SUMO-specific protease 1 [11]. In the present study, we found that the miR-138 expression level was significantly decreased in NSCLC tissues compared to their matched adjacent normal tissues. Besides, it was also downregulated in NSCLC cell lines compared to normal lung epithelial cell. Accordingly, miR-138 may become a biomarker for NSCLC. Moreover, reduced miR-138 expression was tightly associated with the advanced malignancy of NSCLC, suggesting that its downregulation is involved in the malignant progression of NSCLC. In vitro study showed that overexpression of miR-138 significantly inhibited A549 cell growth, invasion and migration, while knockdown of miR-138 enhanced the growth, invasion and migration of A549 cells. These findings suggest that miR-138 acts as a tumor suppressor in inhibiting NSCLC growth and metastasis.

YAP1 is a transcriptional regulator of Hippo signaling [17], and plays important roles in various of human cancers [18]. Wu *et al.* used genome-wide scan of single nucleotide polymorphism, revealing that rs1820453 within the promoter region of YAP1 was associated with small-cell lung cancer survival [19]. Huang et al. showed that miR-497 could inhibit the proliferation of NSCLC by inhibiting the protein expression of YAP1, suggesting that YAP1 plays an oncogenic role in NSCLC. However, evidence in the exact regulatory mechanism of YAP1 expression in NSCLC is still limited. As one gene can be mediated by many miRs, other miRs may be also involved in the regulation of YAP1 expression. In the present study, bioinformatical analysis predicated that YAP1 was a putative target of miR-138. Luciferase reporter assay further confirmed their targeting relationship, and the expression of YAP1 was negatively regulated by miR-138 at the post-transcriptional level in NSCLC cells. Moreover, overexpression of YAP1 markedly reversed the inhibitory effect of miR-138 on NSCLC cell proliferation, but had no effect on NSCLC cell migration and invasion. These findings suggest that YAP1 acts as a downstream effecter of miR-138 in the regulation of NSCLC growth, but may have no affect on NSCLC metastasis. Our results were in consistent with a previous study in oral squamous cell carcinoma cells [20]. Therefore, the miR-138/YAP1 axis may play a common role in regulating the tumor growth in different types of human malignancies. Future studies should focus on the role of Hippo signaling pathway downstream the miR-138/YAP1 axis in NSCLC as well as in other cancer types. In addition to YAP1, several other targets have also been identified such as ZEB2 [21], GIT1 and SEMA4C [22]. Our study expands the understanding of the regulatory mechanism of miR-138 in the regulation of cancer cell proliferation.

Based on the findings in this study, we for the first time suggest that miR-138 inhibits the growth and metastasis of NSCLC cells partly at least via targeting YAP1, suggesting that the miR-138/YAP1 axis may serve as a potential target for the treatment of NSCLC.

## MATERIALS AND METHODS

### Tissue specimens collection

Our study was approved by the Ethics Committee of Hunan Province Tumor Hospital, Changsha, China. NSCLC tissues (n=21) and their matched adjacent non-tumor tissues were collected at Hunan Province Tumor Hospital (Changsha, Hunan, China) from August 2013 to December 2013. The clinical information of these NSCLC patients was summarized in Supplementary Table S1. The written informed consents were obtained. The histomorphology was confirmed by the Department of Pathology, Hunan Province Tumor Hospital. Tissues were immediately snap-frozen in liquid nitrogen after surgical removal and stored at −80°C before use.

### Cell culture and transfection

Four common human NSCLC cell lines (SK-MES-1, A549, H460, and SPC-A1) and a normal human lung epithelial cell line BEAS-2B were purchased from the Cell bank of Central South University (Changsha, Hunan, China). Cells were cultured in DMEM (Life Technologies, Carlsbad, CA, USA) supplemented with 10% FBS (Life Technologies) at 37°C with 5 % CO_2_.

Lipofectamine 2000 (Life Technologies) was used to perform transfection, in accordance with the manufacturer's instruction. YAP1-overexpressing plasmid (Amspring, Changsha, Hunan, China), scramble miR (Amspring), miR-138 mimic (Amspring) and miR-138 inhibitor (Amspring) were diluted with serum-free DMEM, respectively. The diluted Lipofectamine 2000 was then added into the diluted YAP1-overexpressing plasmid, miR-138 mimic, or miR-138 inhibitor. After incubation at room temperature for 20 min, the above mixture was added into the cell suspension, which was then incubated at 37°C, 5% CO_2_ for 6 h. After that, the transfection mixture was replaced by DMEM with 10% FBS. Cells were then cultured for 48 h before the following assays.

### RNA extraction and quantitative real-time PCR

In accordance with the manufacturer's instruction, total RNA was extracted from the tissues and cells by using Trizol reagent (Life Technologies). Quantitative real-time PCR was used to examine the relative miR-138 expression using mirVana™ real-time RT-PCR microRNA detection kit (Life Technologies), in accordance with the manufacturer's instruction. U6 was used as an internal reference. The relative expression of YAP1 mRNA was detected by real-time RT-PCR using the standard SYBR-Green RT-PCR kit (Takara, Otsu, Japan), in accordance with the manufacturer's instruction. GAPDH was used as an internal reference. The specific primers for miR-138 and U6 were purchased from Genecopoeia, Guangzhou, China. The specific primers for YAP1 were shown as follow: Forward, 5′- TAGCCCTGCGTAGCCAGTTA -3′; Reverse, 5′- TCATGCTTAGTCCACTGTCTGT-3′. The specific primers for GAPDH were shown as follow: Forward, 5′- ACAACTTTGGTATCGTGGAAGG-3′; Reverse, 5′- GCCATCACGCCACAGTTTC-3′. The relative expression level was quantified using the 2^−ΔΔCt^ method.

### Dual luciferase reporter assays

The dual luciferase reporter assays were carried out as previous described [23]. In brief, the wildtype YAP1 3′-UTR was constructed by PCR and inserted into the psiCHECK^TM^-2 vector (Promega, Madison, WI, USA). The mutant YAP1 3′-UTR was generated by using Quick-Change Site-Directed Mutagenesis Kit (Stratagene, La Jolla, CA, USA), in accordance with the manufacture's protocol, and then inserted into the psiCHECK^TM^-2 vector. A549 cells were cultured to approximately 70% confluence, and co-transfected with wildtype YAP1-3′UTR or mutant YAP1-3′UTR plasmid (100 ng), and scramble miR or miR-138 mimic (50 nM), using Lipofectamine 2000. After 48 h, dual-luciferase reporter assay system (Promega) was used to determine the activities of renilla luciferase and firefly luciferase. The renilla luciferase activity was normalized to the firefly luciferase activity.

### Western blotting

Western Blotting was carried out as previous described [24]. Briefly, cells were lysed in cold RIPA buffer (Life Technologies). The protein concentration was determined using the BCA Protein Assay Kit (Pierce Chemical, Rockford, IL, USA). Protein was separated with 10% SDS-PAGE, transferred to a PVDF membrane (Life Technologies), and then blocked in 5% nonfat dried milk (Yili, Beijing, China) in DPBS (Life Technologies) for 4 h. The PVDF membrane was then incubated with rabbit anti-YAP1 monoclonal antibody (1:100, Abcam, Cambridge, MA, USA), or mouse anti-GAPDH monoclonal antibody (1:100, Abcam) as an internal reference for 3 h at room temperature, and then washed by DPBS for 10 min. After that, the PVDF membrane was incubated with mouse anti-rabbit secondary antibody (1:20000, Abcam) for 1 h at room temperature. After washing by DPBS for 15 min, the immune complexes on PVDF membrane was detected using the ECL Western Blotting Kit (Pierce Chemical, Rockford, IL, USA). Image-Pro plus software 6.0 was used to analyze the relative protein expression, represented as the density ratio versus GAPDH.

### Cell proliferation, invasion and migration assay

MTT assay was used to examine the cell proliferation as described previously [25]. A549 cells in different groups were plated into a 96-well plate, and cultured at 37°C with 5 % CO_2_ for 12, 24, 48 and 72 h. After that, 20 μL of MTT (5 mg/mL, Life Technologies) was added. After incubation at 37°C for 4 h, 150 μL DMSO was added. After incubation at room temperature for 10 min, the formazan production was detected by determining the optical density (OD) at 570 nm using a Multiskan FC enzyme immunoassay analyzer (Thermo Fisher Scientific).

Cell invasion was examined using the 24-well transwell chambers with a layer of matrigel (Chemicon, CA, USA). For each group, 300 uL of A549 cell suspension, each containing 5000 cells, was added in the upper chamber. DMEM containing 10% FBS was added into the lower chamber. After cultured for 24 h, non-invading A549 cells on the interior of the inserts were removed using a cotton-tipped swab. Invading A549 cells on lower surface of the inserts were stained with 0.1% gentian violet (Sigma, St Louis, Missouri, USA), rinsed by water, and dried in air. Invading A549 cells were observed under a microscope. The cell number was counted.

Wound healing assay was used to examine cell migration. Briefly, cells in different groups were cultured to confluence. Wounds of approximately 1 mm width were created using a plastic scriber. Cells were then washed using DPBS, and cultured in serum-free DMEM for 24h. After that, A549 cells were cultured in DMEM with 10% FBS for 36h. Then, A549 cells were fixed and observed under a microscope.

### Statistical methods

All data in this study are expressed as the mean ± SD of at least three independent experiments. Statistical analysis of differences was performed by one-way analysis of variance (ANOVA) or student t test using SPSS 17.0 software. P value less than 0.05 was considered statistically significant.

## SUPPLEMENTARY FIGURE AND TABLE


